# Multiradiographic Diagnosis of Primary Hepatocellular Carcinoma and Evaluation of Its Postoperative Observation after Interventional Treatment

**DOI:** 10.1155/2022/5292200

**Published:** 2022-08-04

**Authors:** Ning Tang, Jing Zhu, Ying Zeng, Xiao Zhang, Jian Zhou

**Affiliations:** ^1^Department of Radiology, The General Hospital of Western Theater Command, Chengdu, Sichuan 610083, China; ^2^Department of Oncology, The General Hospital of Western Theater Command, Chengdu, Sichuan 610083, China; ^3^Department of Radiology, Joint Security Forces 945 Hospital, Yaan, Sichuan 610083, China

## Abstract

**Objective:**

To investigate the focal imaging performance of MRI and CT multiphase dynamic enhancement scan examination in primary liver cancer patients, analyze its clinical diagnostic value, and provide a basis for early diagnosis of the disease.

**Methods:**

236 patients with primary liver cancer admitted to our hospital from May 2019 to November 2021 were randomly divided into two groups, the control group was given MRI multiphase dynamic enhancement scan diagnostic method, and the observation group was given CT scan combined with the MRI diagnostic method. The patients' examination results and pathological examination results were compared and analyzed, and the therapeutic effects of patients in the two groups after interventional treatment were compared.

**Results:**

After the imaging and pathological examinations of patients in both groups, it was found that the diagnostic accuracy of patients in the observation group and the therapeutic effect after interventional treatment were significantly better than those in the control group.

**Conclusions:**

Compared with CT multiphase dynamic enhancement scan, MRI multiphase dynamic enhancement scan can show multidirectional and multiangle lesions in primary hepatocellular carcinoma patients, with better characteristics of blood supply to hepatocellular carcinoma and a higher accuracy rate.

## 1. Introduction

As one of the malignant tumors, the exact etiology and pathogenesis of primary liver cancer are not clear, but it is generally believed to be related to cirrhosis and viral hepatitis, and its development is also closely related to the patient's living environment [1]. In clinical practice, patients with primary liver cancer need to identify the cause at an early stage and take appropriate treatment measures to improve the efficiency of primary liver cancer disease [2].

The clinical manifestations of primary liver cancer are obviously related to the stage, as follows: (1) Early-stage liver cancer may have no obvious symptoms, or only mild symptoms such as weakness, discomfort, aversion to oil, and nausea. (2) If it is in the middle and late stage, the original liver pain may appear, mostly dull pain or vague pain, which is also the first symptom of primary liver cancer patients. This clinical symptom appears mainly because the growth of the tumor gradually increases the tension of the patient's liver envelope, which is mainly a long-term stabbing or swelling pain. In addition, the clinical symptoms of primary liver cancer patients include weakness, weight loss, abdominal distension, nausea, vomiting, and fever. (3) In the advanced stage, there may also be anemia, jaundice, ascites, lower limb edema, etc. If liver cancer has corresponding metastases, there may also be abnormal clinical manifestations of combined metastases, and advanced liver cancer patients also have anemia, lower limb edema, subcutaneous bleeding, etc. [3]. Patients with advanced hepatocellular carcinoma may also present with anemia, lower limb edema, and subcutaneous bleeding [4]. As the disease progresses, the patient's liver will gradually enlarge, and clinical examination will also reveal irregularly shaped liver margins and nodules on the liver surface as well as masses of various sizes [5]. In the later stages of disease development, cancer cells will metastasize to the lung, bone, and brain, and the metastatic sites will also show corresponding clinical symptoms [6]. Complications in patients with primary liver cancer are mainly manifested as hepatic coma, cancer rupture, and secondary infection [7].

Imaging examinations can examine the occupying lesions in the liver of patients with cirrhosis, thus providing a reference basis for clinical diagnosis and treatment [8]. At present, CT is often used to diagnose cirrhosis with liver cancer, which uses accurate collimated *γ*-rays, ultrasound, X-rays, and highly sensitive detectors to perform cross-sectional scans, with the characteristics of fast scanning speed and clear images, which can better show the intensification characteristics of liver cancer patients [9]. It can display lesions from multiple angles and directions, fully display the blood supply of hepatocellular carcinoma, facilitate the detection of microscopic hepatocellular carcinoma, and does not affect the body significantly [10]. Since both CT and MRI multiphase dynamic enhancement scans can effectively reflect the intensification characteristics of patients with hepatocellular carcinoma, this study aims to further investigate the imaging performance and diagnostic value of MRI and CT multiphase dynamic enhancement scans in patients with cirrhosis and hepatocellular carcinoma in order to provide a basis for early diagnosis of the disease [11].

## 2. Materials and Methods

### 2.1. General Information

The clinical manifestations of these patients included a history of cirrhosis, hepatitis B virus infection, and a persistent increase in fetoprotein, along with wasting, weakness, intermittent epigastric or daring pain, and jaundice of varying degrees [12]. The patients were randomly divided into control and observation groups, with 116 patients in each group, control group: 80 males and 36 females, aged 45 to 80 years and mean age (53.9 ± 5.8) years, and observation group: 76 patients and 40 females, aged 46 to 79 years and mean age (52.6 ± 4.9) years. The differences between the clinical data of the two groups were not statistically significant (*P* > 0.05). The patient information involved in this study has been agreed by the patients, the informed consent form has been signed, and the ethics committee of our hospital approved the study.

### 2.2. Inspection Method

A single MRI diagnosis was given. Four hours before the start of the formal examination, the patient was told not to drink alcohol and to remain in the supine position, entering first by the head, during the examination. In the observation group, patients were given CT scan combined with MRI, and the MRI examination method was the same as that of the control group. Before the start of the CT examination, the medical staff told the patients that they were not allowed to eat or drink 12 hours in advance, and before the start of the formal examination, the patients drank 800 ml of pure water. During the examination, the patient was allowed to breathe steadily and avoid excessive tension, and then the enhanced scan was performed after the routine diagnosis was completed to further improve the accuracy of the diagnosis. The patient's liver was scanned continuously. At the end of the examination, patients diagnosed with primary liver cancer were treated with Philips FD20 CLARITY angiography, and pathological examinations were performed on patients' tumor samples to compare the results of routine and pathological examinations between the two groups, which were also reviewed after treatment.

### 2.3. Observed Indicators

The imaging results and final pathological examination results of the two groups of patients were analyzed and compared, and the compliance rate was calculated; after a period of interventional treatment, whether the scope of the patient's lesion has been reduced during the review process was observed, and the minimum short diameter and maximum long diameter of the patient's tumor were recorded.

### 2.4. Statistical Methods

All data presented in this study were specifically processed and analyzed using the appropriate statistical software. A *t*-test was applied to the processed data, and *P* < 0.05 was considered a statistically significant difference.

## 3. Results

### 3.1. Diagnostic Results

In a specific comparison of the CT and MRI results with the patient's pathological diagnosis and the compliance rate, it can be concluded that the number of compliance of CT examination results is 44 and the compliance rate is 88%, while the number of compliance of MRI examination results is 48 and the compliance rate is 96%, and the difference between these two examination methods is statistically significant (*P* < 0.05, see Table 1). Therefore, in the postoperative evaluation of TACE for hepatocellular carcinoma, MRI is the best choice.

### 3.2. Treatment Effect after Intervention in Two Groups of Patients

After a period of intervention in both groups, the patients' treatment effects were evaluated by applying the pretreatment clinical diagnostic methods, and it was found that the scope of lesions in both groups was significantly reduced, and the difference between the minimum short diameter of tumors in the control group and the observation group is statistically significant (*P* < 0.05) (see Table 2).

### 3.3. Surgical and Pathological Findings

The maximum diameter of the masses ranged from 1.0 to 13.0 cm, with a mean value of (6.5 ± 3.8) cm. 7 of the masses were grayish white, and 3 were grayish yellow with clear borders. The other two lesions were smaller and no cystic changes or necrosis was observed. Immunohistochemistry showed positive staining for synaptophysin (Syn), chromogranin A (CgA), CD56, and CK19, which are characteristics of neuroendocrine carcinoma (Table 3).

### 3.4. Location and Size of Lesions and Number of Lesions

A total of 10 lesions were detected by CT and MRI, consistent with the surgical pathology; 5 lesions were detected by CT and 7 lesions were detected by MRI (2 cases were examined by both CT and MRI); 6 lesions were found in the right lobe of the liver (60%) and 2 in the left lobe of the liver (20%), and 2 lesions were larger than the junction area of the left and right lobes (20%); 4 lesions were ≤3 cm, 5 lesions were between 3 and 10 cm, and 1 lesion was >10 cm.

### 3.5. CT and MRI Findings

In 7 patients, no cirrhotic background was seen in the liver, and the lesions appeared as lobulated masses or round-like nodular foci, 8 lesions showed internal liquefied necrosis or cystic lesions, and 2 lesions did not show cystic lesions and necrosis. The MRI showed the following results: 5 lesions showed T1WI low signal and T2WI and DWI high signal (Figure1), the center of the lesion had T1WI lower signal and T2WI higher signal shadow, suggesting partial cystic degeneration or liquefied necrosis, 3 lesions in the arterial phase had heterogeneous enhancement (Figure 2), and the other two lesions were smaller, 1.0 cm and 1.3 cm in diameter, with no cystic degeneration or necrosis, and were significantly strengthened in the arterial phase (see Figures 3 and 4).

## 4. Discussions

In China, most imaging tools, such as CT and MRI, are used to evaluate the efficacy of hepatocellular carcinoma after TACE. MRI, ultrasound, and CT are mostly used for clinical diagnosis, and some scholars believe that CT and MRI examinations can improve the detection rate of hepatocellular carcinoma and have a higher diagnostic value for patients with microscopic hepatocellular carcinoma [13, 14]. CT and MRI multiphase dynamic scans show the intensification characteristics of patients with hepatocellular carcinoma, in which the arterial phase intensification is obvious and can present high signal characteristics, and normal liver parenchyma is mostly nonenhanced and lightly intensified [15]. The degree of liver parenchyma enhancement can reach the peak, and after reaching the peak, the patient's lesion shows iso- and low-signal status and the lesion density decreases in the delayed phase, and patients with hepatocellular carcinoma can fully demonstrate the “fast-in and fast-out” enhancement characteristics [16]. The results of this study showed that when multiphase dynamic enhancement scans were performed by CT and MRI, patients with MRI showed high signal in the arterial phase and iso- and low signal in the portal and delayed phases, which could show the “fast-in and fast-out” characteristics [17]. This indicates that patients with cirrhosis with hepatocellular carcinoma have a high detection rate of foci by CT and MRI in clinical diagnosis [18].

The pathological features of hepatocellular carcinoma can show different degrees of pseudoenvelope, presenting a dual structure with a thin inner layer and relatively abundant compressed blood vessels and new bile ducts in the outer layer of the envelope [19]. The accuracy of CT multiphase dynamic scan is determined by the difference in density between lesion enhancement and normal liver parenchyma, and its enhancement characteristics are mostly shown within a short time of contrast injection, which may not be the best time period for tumor display, and it has radioactive damage, and repeated examination may damage the patient's organism; MRI multiphase dynamic enhancement scan is done according to the occurrence of lesion site [20]. MRI multistage dynamic enhancement scan can show the lesion in multiple directions with selective scans in the coronal plane, cross-sectional plane, and even angular oblique scans according to the occurrence of the lesion, which is more sensitive for the diagnosis of microscopic hepatocellular carcinoma and has higher localization accuracy than CT examination [12].

After interventional treatment of patients with hepatocellular carcinoma, specific deposition of iodine oil can be observed as it is deposited within and around the tumor lesion to understand the changes in size and number of lesions in the liver before treatment, involvement of portal veins, metastases in the surrounding organs, and the form of iodine oil deposition [21]. In general, if the iodine oil deposits are dense and evenly distributed, the tumor necrosis rate will be high, while the tumor survival rate will be high in the areas with fewer or even no iodine oil deposits [22]. Plain CT scan can reflect the specific changes after tumor treatment, such as necrosis, liquefaction, fibrosis, cystic changes, new lesions, and the presence of surviving tumor tissue [23, 24]. Enhanced dual-light scans allow clearer visualization of the eastern part of the vegetative scan and specifically reflect the blood supply of new lesions and residual tumor tissue [25].

In conclusion, MRI can very accurately assess the efficacy of post-TACE tissues for hepatocellular carcinoma. Therefore, MRI is the best choice for post-TACE evaluation of hepatocellular carcinoma.

## Figures and Tables

**Figure 1:** Axial MRI images of a patient with HCC in the right lobe of the liver. (a) A T2 high signal nodule is seen in the right posterior lobe of the liver. (b) The lesion is mostly isosignal on in-phase T1 images, with slightly higher signal (arrows) locally. (c) The lesion is significantly low signal (arrows) on in-phase T1 images, suggesting that the lesion contains lipid. (d) The lesion is significantly enhanced in the arterial phase. (e) Delayed phase contouring.

**Figure 2:** Axial MRI images of a patient. (a) A T1 low signal is seen in the left lobe of the liver; (b) a T2 high signal mass shadow with multiple high signals (arrows) on T1WI and a slightly high center surrounded by a low signal ring (arrows) on T2WI is seen in the mass, suggesting intranodal hemorrhage; (c) arterial phase mass enhancement; (d) delayed phase contouring.

**Figure 3:** Axial MRI image (pulmonary enhancement) of a patient with HCC in the hepatic parietal region. (a) T1 low signal in the hepatic parietal region; (b) T2 slightly high signal nodule; (c) marked enhancement in the arterial phase; (d) portal venous phase; (e) transitional phase; (f) hepatobiliary phase contouring with a distinct low signal ring around the nodule (d–f triangle).

**Figure 4:** Axial MRI images of a patient with HCC in the left lobe of the liver. (a) A T2 mixed slightly high signal mass is seen in the left lobe of the liver; (b) significant inhomogeneous enhancement in the arterial phase; (c) contouring and separation in the portal vein phase (arrows).

**Table 1:** Diagnostic compliance rate.

Group	Number of cases	Diagnostic method	Diagnostic coincidence number	Coincidence rate
Experience group	60	MRI	48^*∗*^	95%^*∗*^
Control group	60	CT	45	89%
*P* value	<0.05	<0.05		

Note: ^*∗*^Significant difference; *P* < 0.05, statistically significant.

**Table 2:** Treatment results of patients in both groups after intervention $\left(\bar{x}\pm s\right)$.

Group	Number of cases	Minimum short diameter	Longest diameter	Enhancement zone score in the residual arterial phase
Experience group	116	1.02 ± 0.24	3.38 ± 0.22	4.35 ± 0.45
Control group	116	1.56 ± 0.65	3.78 ± 0.54	4.52 ± 0.54
*t*	—	7.36	0.32	0.32
*p*	—	0.02	0.86	0.87

**Table 3:** Clinical manifestations and immunohistochemistry of PHNEC patients.

Serial number	Age	Gender	Tumor location	Number of tumors	Maximum diameter of tumor (CM)	Clinical manifestation	Immunohistochemistry			
							Syn	CgA	CD56	CK19
1	74	Female	Junction of left and right lobes	1	12.8	Middle and upper abdominal distention and pain	+	+	+	+

2	25	Male	Junction of left and right lobes			Physical Findings Physical Findings	+	+	+	+

3	45	Male	Left lateral lobe	1	1.5	Right upper abdominal distention and pain	+	+	+	+

4	81	Female	Right posterior lobe	1	7.4	Physical Findings Physical Findings	+	−	+	+

5	75	Male	Right anterior lobe	1	3.1	Middle and upper abdominal distention and pain	−	+	+	−

## Data Availability

The experimental data used to support the findings of this study are available from the corresponding author upon request.
